The article "Necrosis of the 4th and 5th Digits after Intra-Articular Injection of Diazepam into the Wrist" was published in 2011. Journal: Case Rep Surg.

# Necrosis of the 4th and 5th Digits after Intra-Articular Injection of Diazepam into the Wrist

**DOI:** 10.1155/2011/347523

**Published:** 2011-09-14

**Authors:** Niklas Iblher, Gerd Bjoern Stark, Vincenzo Penna

**Affiliations:** Department of Plastic and Hand Surgery, University of Freiburg Medical Center, Hugstetter Straße 55, 79106 Freiburg, Germany

## Abstract

A 75-year-old woman presented with progressing pain, cyanosis, and hypaesthesia in her left hand after an intra-articular injection with diazepam into the wrist for osteoarthritis-related pain. Due to an iatrogenic intra-arterial injection, malperfusion of the ulnar digits developed. Angiography revealed blockage of perfusion of the 4th and 5th digits. Despite intra-arterial lysis, heparinisation, and vasodilatation, perfusion could not be reinstalled. Necrosis of the distal phalanges of the 4th and 5th digits developed, which had to be treated with amputation. The pathomechanism of tissue damage and the treatment options after intra-arterial injections are reviewed and discussed.

## 1. Case Report

A 75-year-old woman (nonsmoker with history of hypertension and depression) had repeatedly been administered an intra-articular injection with diazepam for left-sided chronic wrist pain due to osteoarthritis by a primary physician and chiropractor. After the last injection, she immediately developed progressing, cyanosis and hypaesthesia pain in her hand (Figure 1). The symptoms became unbearable after 3 days and the patient presented to our institution. After immediate admission digital angiography showed a complete blockage of perfusion to her 4th and 5th left fingers (Figure 2). Intra-arterial lysis therapy with urokinase was initiated but only slightly improved arterial flow in the ulnar digital artery of the 5th digit in the control angiography and was discontinued after 2 days due to an increasing hematoma on the upper arm. Intravenous heparinisation was administered from the day of hospitalization, and vasodilatation with prostaglandin was started on the second day. Both medications were continued until day 9 when an inhibition of platelet aggregation was started with aspirin 100 mg and clopidogrel 75 mg daily. CK was elevated from 481 U/l on day 3 to 642 U/l on day 5. The patient was discharged on the following day after a total of 10 days of hospitalization. During this time, the cyanotic 4th and 5th digits showed some improvement and the pain and hypaesthesia resolved. The patient was followed up as an outpatient for a total of 5 weeks during which time the acral areas of the digits progressed into dry necrosis (Figure 3). With no further treatment option left, the 4th digit was amputated at the distal middle phalanx and the 5th digit was exarticulated in the distal interphalangeal joint.  Figure 4 shows the intraoperative view of a thrombosed digital artery in the 5th digit. Wound healing was uneventful. Histological workup of the amputated tissue showed necrotic soft tissue and bone, a mildly active osteomyelitis, and small vessel thrombosis.  Figure 5 shows the result 2 weeks postoperatively.

The patient denied to name the primary physician because she “has always been treated so well.” 

## 2. Discussion

Distal gangrene of extremities after intra-arterial injections has been described in the literature before, most commonly in i.v. drug abusers or after arterial catheterization [1]. While intra-articular injection of various drugs in i.v. drug abusers has become a common problem [2–5], the sequelae are still difficult to prevent and often catastrophic. Intra-arterial injection of diazepam in convulsive patients have also been described [6].

To our best knowledge, this is the first report of a case of iatrogenic, intra-arterial injection resulting from a failed “therapeutic” intra-articular injection of diazepam by a medical professional for osteoarthritis-related pain. While the oral application of diazepam as an adjunct medication for rheumatoid arthritis has been described [7, 8], we consider intra-arterial injection of diazepam as medical malpractice exposing the patient to unnecessary risks which in the present case resulted in serious sequelae. Diazepam as a long-lasting benzodiazepine does not have any analgetic or anti-inflammatory effect that could prove beneficial in this clinical setting, thus we have to classify this treatment as medical malpractice exposing the patient to unnecessary risks with like in this case catastrophic sequelae. 

The pathomechanism of peripheral gangrene after intraarterial injections is yet poorly understood. Many theories have been put forward including inflammation of the endothelium [9, 10], liberation of vasoactive amines [11], mechanical blockage of the microcirculation [12, 13], or a penetration of the plasma membrane of the mostly lipophilic substances with consequent lysis [14]. All concepts seem to agree on a final mechanism of peripheral underperfusion due to endarteritis, vasospasm, and thrombosis leading to tissue necrosis.

Consequently, numerous treatment options addressing the proposed mechanisms have been suggested. Most authors agree on consequent analgesia, early mobilization of the extremity, and administration of i.v. heparin, although understandably in most reports there is no control group to this approach, proving that heparin is really responsible for at least partial resolution of underperfusion. Elevation may be harmful when perfusion pressure is low but edema leading to compression of small vessels is also harmful. The optimal position may be the one that gives most pain relief, whether it is slightly lowering or elevating the hand. Thrombolysis (streptokinase [2], rt-PA [5, 15], and urokinase [16]) has been suggested in early stages and seems to show at least partial success in some cases 

Vasodilatation using different substances (prostaglandins [5, 15, 17], papaverine [16], tolazoline [2], reserpine, or nitroglycerin [18]) is applied to address the vasospasm.

A sympatholytic and therefore also vasodilating effect is achieved by stellate ganglion blocks or axillary plexus anesthesia [16, 19]. Plexus anesthesia has an additional analgetic benefit. 

Dextrans [19] and aspirin, usually starting on day 4-5, have also been proposed [20]. Application of high-dose systemic corticosteroids is part of some treatment schemes [20]. Hyperbaric oxygen therapy has been reported to have an effect on the malperfused areas by Adir et al. [21] but failed to show effect in the report from Chang and Lin [22].

Like in most medical fields the existence of so many treatment options suggests that none shows reliable and satisfying results for this difficult condition. The resultant tissue necrosis can only be handled by excision and amputation. In necrotic fingers without any signs of inflammation, we suggest to wait for at least 4 weeks before definitive amputation to allow for clear demarcation, thus preventing unnecessary secondary intervention after insufficient resection or exaggerated resections of healthy tissue.

## 3. Conclusion

This case report should remind us of the fact that injections around the wrist carry the risk of intra-arterial injections with possibly catastrophic results. Based on the frequency of reports in the literature, this condition is not as rare as one might think. Yet, there is still no clear understanding of the mechanisms leading to peripheral gangrene and consequently there is no reliable treatment available.

Intra-articular diazepam injections for osteoarthritis-related pain is an absurd concept in our view and although “it is only” an injection that can lead to severe complications.

## Figures and Tables

**Figure 1:** Clinical findings after admission of the patient, 3 days after the injection.

**Figure 2:** Digital angiography showing complete blockage of perfusion to the 4th and 5th digits.

**Figure 3:** Demarcated necrosis of the 4th and 5th fingers after 5 weeks.

**Figure 4:** Intraoperative view of the amputated 5th finger showing a thrombosed digital artery (circle) with the visible thrombus at the dissected end (arrow).

**Figure 5:** Amputated fingers after suture removal 2 weeks postoperatively.
